# PD-1 Coexpression Gene Analysis and the Regulatory Network in Endometrial Cancer Based on Bioinformatics Analysis

**DOI:** 10.1155/2021/9923434

**Published:** 2021-05-25

**Authors:** Lina Wang, Zhen Liu, Wenwen Zhang, Aihua Zhang, Pengpeng Qu

**Affiliations:** ^1^Third Central Hospital of Tianjin, Tianjin, China; ^2^Tianjin Key Laboratory of Artificial Cell, China; ^3^Artificial Cell Engineering Technology Research Center of Public Health Ministry, Tianjin, China; ^4^Tianjin Institute of Hepatobiliary Disease, Tianjin, China; ^5^Department of Gynecology, Chifeng Municipal Hospital, Chifeng Clinical Medical School of Inner Mongolia Medical University, Chifeng, China; ^6^Tianjin Central Hospital of Gynecology and Obstetrics, Tianjin, China

## Abstract

Gynecological malignancies are tumors of the female reproductive system, mainly cervical cancer, endometrial cancer, and ovarian cancer. Endometrial cancer (EC) is the most common gynecological malignant tumor in developed countries. The aim of this study was to construct a network of programmed cell death protein 1 (PD-1) coexpressed genes through bioinformatics analysis and screen the potential biomarkers of PD-1 in endometrial cancer. In addition, genes and pathways involved in PD-1 and modulating tumor immune status were identified. We select the EC transcriptomic dataset in TCGA to retrieve gene sets on the cBioPortal platform, and the PD-1 coexpressed genes were obtained on the platform. GO and KEGG enrichment analysis of coexpressed genes was performed using the DAVID database. The target protein-protein interaction (PPI) network was constructed using Cytoscape 3.7.1 software, and the hub genes were then screened. A total of 976 coexpression genes were obtained. The enrichment analysis showed that PD-1 coexpressed genes were significantly enriched in overall components of the cell structure, the interaction of cytokines with cytokine receptors, chemokine signaling pathways, and cell adhesion molecules (CAMs). Ten hub genes were obtained by node degree analysis. CD3E gene is involved in the prognosis and immune process of EC, and the expression level is related to PD-1 (Pearson correlation coefficient is 0.82, *P* < 0.01). Patients with low CD3E gene expression in EC have a poor prognosis. The coexpression hub genes of PD-1 are related to immunity, in which CD3E is a prognostic marker that is involved in the PD-1/PD-L1-induced tumor immune escape. This study provides a new area to study the mechanism of PD-1/PD-L1 in EC and the precise treatment with targeted drugs.

## 1. Introduction

Gynecological malignancies are tumors of the female reproductive system, mainly cervical cancer, endometrial cancer, and ovarian cancer. Endometrial cancer is the most common gynecological malignant tumor in developed countries [1]. Although people continue to improve the existing treatment methods to improve the effect of surgical treatment, combined with chemotherapy and radiotherapy-based auxiliary treatment methods, the treatment effect and disease prognosis are still not satisfactory. In recent years, with the importance of the concept of the tumor microenvironment and the continuous deepening of research on the tumor immune mechanism, the role of tumor immunotherapy in the treatment of malignant tumors has been increasing.

The goal of immunotherapy is usually to reverse the immune escape mechanism of tumors and restore the local immune response against cancer cells [2, 3]. Recent immunotherapy research focuses on antibodies that block programmed cell death protein 1 (PD-1) or its ligands (such as PD-L1). The combination of PD-L1 and PD-1 can cause T cell dysfunction and failure and promote the production of IL-10 in tumors and thus promote T cell apoptosis [4]. Some scholars have found that PD-1 is significantly expressed in peripheral blood of patients with liver cancer, kidney cancer, and gastric cancer [5], and the expression level of PD-1 on T cells may be positively correlated with the progression of gastric cancer and chronic lymphocytic leukemia [6, 7]. Since the first PD-1/PD-L1 inhibitor (pembrolizumab) was approved by the Food and Drug Administration in 2014, many immune checkpoint inhibitors have been used in clinical practice [8]. PD-1/PD-L1 has shown effective and long-lasting antitumor effects on inhibitors, especially in some refractory tumors [9, 10]. Although PD-1/PD-L1 inhibitors have still attracted widespread attention, their relatively low response rate has limited their use in patients [11, 12]. In addition, some patients still show resistance and related adverse reactions. There is a need for high-sensitivity assays or comarkers for identifying biomarker expression in patient populations to identify more precise targets for PD-1/PD-L1 and improve the feasibility of treatment. The urgent problem is to improve the accuracy and effectiveness of PD-1/PD-L1 inhibitors in EC treatment. At the same time, it also helps to understand the PD-1/PD-L1 pathway regulation mechanism in EC more clearly and deeply. In addition, PD-1/PD-L1 therapy can also be combined with other therapies (such as chemotherapy and targeted therapy), which is expected to achieve the purpose of improving efficacy, reducing side effects, and improving patient survival and quality of life.

The purpose of this study was to analyze the EC dataset in The Cancer Genome Atlas (TCGA) database (https://cancergenome.nih.gov/) using bioinformatics methods, which will help to screen and analyze PD-1 coexpressed genes, describe the PD-1 molecular regulatory network, explore the possible involvement of PD-1 in EC biological processes and core genes related to prognosis, and provide new clues for EC anti-PD-1 research.

## 2. Materials and Methods

### 2.1. Materials

The dataset downloaded from this study is from the TCGA database, a research project of the National Cancer Institute, which uses a consistent genomic platform to analyze at least 20 different tumor types and provide researchers with original and processed data [13]. cBioPortal is one of the TCGA online data analysis platforms, which contains genetic mutations and transcriptome and proteomics data. In this study, the EC dataset in the TCGA database was selected on the cBioPortal platform. There were 549 clinical samples, including 177 RNA-seq samples.

### 2.2. PD-1 Expression in EC

Dynamic analysis of PD-1 gene expression profile data was performed through the GEPIA (http://gepia.cancer-pku.cn/) website to obtain the PD-1 expression level and survival analysis results in EC tissues.

### 2.3. Data Processing and PD-1 Coexpression Gene Screening

The data of 177 RNA-seq samples were statistically analyzed through the cBioPortal platform, and information on PD-1 coexpressed genes was obtained. The screening criteria for genes with coexpression relationship were Spearman coefficient > 0.3.

### 2.4. Function and Enrichment Analysis

The DAVID database (https://david.ncifcrf.gov/summary.jsp) was used to perform GO function enrichment and KEGG pathway enrichment analysis of PD-1 coexpressed genes. DAVID is an online bioinformatics resource designed to provide researchers with a comprehensive set of functional annotation tools to understand the biological mechanisms involved in the function of a large number of genes or proteins [14]. A *P* value of <0.05 and the number of genes greater than 10 represent statistically significant results.

### 2.5. Construction of PPI Network and Hub Gene Screening

The STRING database [15] (https://string-db.org) and Cytoscape 3.7.1 software [16] were used to jointly construct a protein-protein interaction (PPI) network for PD-1 coexpressed genes. The STRING database integrates a text library, experimental/biochemical evidence, coexpression data in PubMed, and database correlations, thereby providing an interactive analysis platform where proteins can be evaluated for connections, associations, and interactions. The Cyto-ubba plug-in is based on the top 10 genes with the highest degree as core genes. 10 hub genes and PD-1 genes were introduced for interaction analysis in the STRING database online analysis platform, an interaction analysis network was established between hub genes and PD-1, and the interaction between hub genes and PD-1 was described.

### 2.6. Survival Analysis

Combined with the clinical information of EC, the gene expression of hub (transcripts per million (TPM)) was grouped on the GEPIA website, and the quartile method was used to separate the high expression group (≥75%) and the low expression group (≤25%). These hub genes were analyzed for survival using the logrank test and Kaplan-Meier test. The logrank test results *P* < 0.05 considered the differences to be statistically significant, and then, coexpressed genes related to the prognosis of EC were screened.

### 2.7. Correlation Analysis between Prognosis-Related Hub Genes and PD-1

The 10 hub genes were analyzed on the GEPIA website, and the hub genes related to the prognosis of EC were screened, and their correlation with PD-1 expression was analyzed and plotted.

## 3. Results

### 3.1. PD-1 Expression in Endometrial Cancer and Its Impact on Prognosis

The difference in PD-1 expression between endometrial cancer and normal tissues in the TCGA database was analyzed on the GEPIA website. The results showed that compared with normal tissues, PD-1 expression was significantly increased in EC. In addition, the overall survival time of patients with high expression of PD-1 EC was significantly higher than that of patients with low expression.

### 3.2. PD-1 Coexpression Gene Screening and Enrichment Analysis

Coexpressed genes of PD-1 gene were screened on the cBioPortal platform, and there were 976 coexpressed genes. The GO enrichment analysis of the coexpressed genes showed that the coexpressed genes were mainly concentrated in biological processes such as protein binding, cytoplasmic membrane, cell membrane and plasma membrane components, and cell structure (Figure 1(a)). KEGG enrichment analysis showed that PD-1 coexpressed genes were significantly enriched in the interaction of cytokines with cytokine receptors, chemokine signaling pathways, and cell adhesion molecules (CAMs) as seen in Figure 1(b).

### 3.3. PPI Network Construction and Interaction Analysis of Coexpressed Genes

The STRING database shows that there are 5384 pairs of interactions between these coexpressed genes, which are much higher than the expected value of 532, and the average node degree is 33.9. The top 10 genes with the highest degree are CD2, PRF1, CTLA4, TBX21, CD3E, CCR5, CXCR3, LCK, IL2RG, and CD247. These genes occupy an important position in the entire network structure. 10 hub genes and PD-1 genes are introduced to the STRING database online analysis platform, and an interaction analysis network was established between hub genes and PD-1 (Figure 2). The results show that the hub genes that interact with PD-1 are CD2, PRF1, CTLA4, TBX21, CD3E, CCR5, CXCR3, LCKH, and CD247. CD3E is an important gene related to the prognosis of EC. CD3E gene is involved in the immune process, and its expression is related to PD-1 (Pearson correlation coefficient is 0.82; *P* value is less than 0.01). Those with low CD3E gene expression in EC have a poor prognosis.

### 3.4. Hub Gene Survival Analysis

On the GEPIA website, using the EC data available on the platform, the hub genes of the top 10 degrees were analyzed for survival. The results showed that among EC patients, only the expression level of CD3E gene was different from the overall survival time of EC patients. Compared with normal tissues, CD3E expression was significantly increased in EC (Figure 3(a)), and EC patients with high CD3E gene expression had a better prognosis than the CD3E gene low expression group (Figure 3(b)). CD3E gene is involved in the immune regulation of cells. Defects in this gene lead to immune deficiency and may be important genes related to the prognosis of EC.

### 3.5. Correlation Analysis of CD3E Gene and PD-1

The correlation between the expression of CD3E gene and PD-1 in EC was analyzed on the GEPIA platform (Figure 4). The Pearson correlation coefficient of CD3E gene and PD-1 was 0.82, and the *P* value was less than 0.01, indicating that this gene not only was related to the prognosis of EC but also has a coexpression relationship with PD-1. In EC, CD3E gene may be involved in the PD-1/PD-L1-mediated tumor immune escape process.

## 4. Discussion

In recent years, immunotherapy has become a promising cancer treatment, which has shown a lasting response in some patients. PD-1/PD-L1 as a target for cancer immunotherapy has shown clinical therapeutic value in a variety of tumors. PD-1/PD-L1 inhibitors are currently in phase II clinical trials for advanced endometrial cancer. One patient had disease progression after the previous three chemotherapy treatments and had a complete remission (CR) of up to 17 months after receiving pembrolizumab [17]. Twenty-four patients with endometrial tumor tissue or mesenchymal cells with PD-L1 expression ≥ 1% in immunohistochemical staining participated in a phase Ib clinical trial (NCT 02054806), indicating that pembrolizumab has tolerable drug toxicity and is resistant to treatment. The follow-up of the effect found that the objective response rate (ORR) was 13% (3/24) and stable disease (SD) was 13% (3/24) of the treatment [18]. The response rate of patients in the Mumizumab-treated group was 13%, and most of the tumor patients were ineffective in anti-PD-1/PD-L1 treatment. All these suggest that the role of the PD-1/PD-L1 pathway in EC and the network regulation mechanism need to be further studied in order to obtain more accurate and effective antitumor effects.

In this study, TCGA's EC dataset was analyzed, and 976 genes coexpressed with PD-1 were screened from the transcriptome data. These genes are mainly enriched in integral components of the plasma membrane such as the cytoplasmic membrane and cell membrane and participate in the interaction of cytokines and cytokine receptors and cell adhesion molecules (CAMs). The chemokine signaling pathway may play a role in cellular immune regulation and signal transfer and may be involved in the immune escape mediated by the PD-1/PD-L1 pathway. Network interaction analysis of PD-1 coexpressed genes revealed that 10 genes had the most extensive effects with other genes. Gene annotation of these genes found that they are involved in the immune response and play an important role in the immune response. Among them, CD2, CTLA4, LCK, TBX21, CD247, and CD3 are related to T cell development and maturation, functional regulation, and signaling functions and play a vital role in adaptive immune response. CTLA4 is a negative regulator of T cells and can control T cell activation by competing with the costimulatory molecule CD28 for binding to the shared ligands CD80 and CD86. Some scholars have found that patients with stage IV endometrial cancer with mismatch repair defects and PD-L1 negative stage show a strong clinical response to the combined inhibition of PD-1 and CTLA-4 [19]. Lymphocyte-specific protein tyrosine kinase (LCK) signaling regulates cisplatin resistance and induces DNA repair genes. Targeting LCK signaling through the immunosuppressive drug saracatinib, which is currently undergoing clinical evaluation, can make chemoresistant tumor cells sensitive to cisplatin and provide opportunities for targeting signaling pathways in endometrioid tumors [20]. The function of CD247 enhances the T cell antigen receptor (TCR) signaling cascade. Defects in CD247 function can cause TCR to participate in impaired T cell activation. Some scholars have shown that compared with patients with ovarian cysts, the expression of CD247 in peripheral blood lymphocytes of patients with ovarian cancer is reduced, while the expression of CD247 in tumor-infiltrating lymphocytes of cancer tissues is reduced compared to adjacent tissues, and the abnormal expression of CD247 is related to differentiation and classification of ovary cancer. This finding suggests that CD247 targeted therapy could be a potential treatment strategy for ovarian cancer. CXCR3 is a receptor for C-X-C chemokines CXCL9, CXCL10, and CXCL11. It mediates the proliferation, survival, and angiogenic activity of human mesangial cells (HMCs) through the heterotrimeric G protein signaling pathway and may promote cell chemotaxis. Studies have found that changes in the expression level of CXCR3 are closely related to endometriosis and endometrial cancer and provide help for the differential diagnosis of endometrial cancer [21]. The IL2RG gene is located on the X chromosome and is mutated in humans with X-linked severe combined immunodeficiency (XSCID). IL2RG controls lymphocyte development, growth, differentiation, and survival and is associated with allergic and autoimmune diseases, cancer, and immune deficiency [22]. PRF1 (perforin-1) plays an important role in killing other cells recognized by the immune system as nonself. Some scholars have reported that the expression of perforin in CD8^+^ tumor-infiltrating lymphocytes and peripheral blood T lymphocytes in patients with endometrial cancer increases the cytolytic capacity of CD8^+^ T cells [23]. CCR5 is a cell membrane protein that is a member of the G protein-coupled receptor (GPCR) superfamily. Both CCL5/CCR5 axis and CCL3/CCR5 axis may be involved in the migration and proliferation of oral cancer cells [24]. The STRING network interaction analysis of the hub gene and PD-1 showed that except for the IL2RG gene, the remaining nine hub genes interacted with PD-L1. It is speculated that these nine hub genes in the PD-1/PD-L1 pathway play an important role. Further analysis of the survival of 10 hub genes revealed that among EC patients, only the CD3E gene was associated with the prognosis of EC, and the prognosis in the high expression group was better than that in the low expression group.

CD3 is a T cell coreceptor complex and is essential for TCR signaling and T cell differentiation. The CD3 complex consists of four transmembrane proteins, *δ*, *γ*, *ε*, and *ζ*. Abnormal expression of any of these proteins has been found to be associated with immunodeficiency diseases [25]. CD3E is a member of the CD3 complex, which exists on the surface of T lymphocytes and plays a vital role in the adaptive immune response. Studies have shown that although the expression of PD-L1 in tumor biopsy tissue can indeed predict the response to anti-PD-1 treatment, many tumors predicted to be PD-L1 positive do not respond, and there are also in PD-L1 negative tumors some reactions [26, 27]. Therefore, some scholars examined the correlation between CD3E expression and putative targets in 9,601 human tumors spanning 31 cancer types. In a dataset of 26 patients receiving anti-PD-1 treatment, CD3E and the coexpression of PD-1 were higher than that of nonresponders. Some patients with a high correlation of CD3E-PD-1 did not respond, while other patients with low correlation did respond to anti-PD-1 treatment. When examining anti-PD-1 responders and nonresponders in metastatic melanoma, scholars found a significantly higher correlation between CD3E and PD-1 between responders and nonresponders, which supports the tumor hypothesis related to CD3E expression in the microenvironment [28]. That can be used as a useful criterion for identifying new therapeutic targets with potential for therapeutic response. Similarly, in a similar analysis of clear cell renal cancer patients' response to immune checkpoint therapy, no significant difference in CD3E-PD-1 correlation was found between responders and nonresponders [29]. More detailed expression analysis of responders and nonresponders in other cancer types will help elucidate other genetic and tumor microenvironmental factors that influence the response to new and existing therapies [29, 30]. We believe that CD3E may be expressed in T cells in the tumor microenvironment and is a promising therapeutic target. The high expression of CD3E in this study is a favorable prognostic factor in EC, and it is related to the occurrence and invasion of EC. CD3E may become a biomarker to evaluate the prognosis of EC anti-PD-1 therapy. The prediction of disease and the prognosis are of certain clinical significance.

The limitation of this study is that further research is still needed to verify our findings. In addition, functional research on the screened genes needs to be explored.

## 5. Conclusions

PD-1 as an important molecular target for tumor immunotherapy plays an important role in the antitumor treatment of EC. In this study, by analyzing the EC dataset in TCGA, the coexpressed CD3E gene of PD-1 related to the prognosis of EC was screened, and their regulatory network was analyzed, which provided a new reference for the anti-PD-1 research of EC.

## Figures and Tables

**Figure 1:** (a) The significantly enriched KEGG pathways of coexpression genes. (b) The significantly enriched GO biological processes of coexpression genes.

**Figure 2:** The protein-protein interaction analysis of PD-1 and hub genes.

**Figure 3:** (a) Expression differences between endometrial cancer and normal tissues. Note: ^∗^*P* value < 0.01. (b) Survival analysis of CD3E in EC patients.

**Figure 4:** Analysis of the relationship between the expression of CD3E protein and PD-1 protein.

## Data Availability

The data generated during the present study are available from the corresponding author on reasonable request.

## Abbreviations

TCGA: The Cancer Genome Atlas
DAVID: Database for Annotation, Visualization, and Integrated Discovery
KEGG: Kyoto Encyclopedia of Genes and Genomes
GO: Gene Ontology
PD-1: Programmed cell death protein 1
EC: Endometrial cancer
PPI: Protein-protein interaction
CAMs: Cell adhesion molecules.
